RETRACTED

# The Inflammasome NLRC4 Protects against Cryptococcus gattii by Inducing the Classic Caspase-1 to Activate the Pyroptosis Signal

**DOI:** 10.1155/2022/7355485

**Published:** 2022-03-16

**Authors:** Yongbin Wang, Feifei Feng, Hui Wang, Ying Zhang, Yuqing Chen

**Affiliations:** ^1^Department of Respiratory Medicine, The Second Hospital, Cheeloo College of Medicine, Shandong University, Jinan, Shandong 250033, China; ^2^Cheeloo College of Medicine, Shandong University, Jinan, Shandong 250033, China; ^3^Department of Respiratory Medicine, First Affiliated Hospital of Bengbu Medical College, Bengbu, Anhui 340300, China

## Abstract

*Cryptococcus* is one of the most pathogenic invasive fungi, and its interaction with the host's natural immunity, especially the role of the inflammasome family, has not been fully elucidated. As an important member of the inflammasome family, NOD-like receptor (NLR) family caspase recruitment domain (CARD) containing 4 (NLRC4) has been proven to protect lungs from damage from a variety of pathogens. In this study, we investigated the protective effect and mechanism of NLRC4 on cryptococcal pulmonary infection using NLRC4-/-mice in vivo and NLRC4-/-macrophages in vitro models stimulated by cryptococcal cells. We apply small animal fluorescence imaging to detect the fungal burden in the lungs and living body micro-CT scans of mice and in vitro tissue micro-CT scans to compare differences in infection foci nodules and histopathological lesions, and the activation of caspase-1 and downstream cytokines were detected by Western bolt and ELISA, etc. The results demonstrated that cryptococcal infection can activate the Nod-like receptors of caspase-1 activation and NLRC4 inflammasomes in macrophages and dendritic cells and affect downstream IL-1*β* and IL-18 release. After cryptococcal infection, the survival rate, lung fungal burden, and histopathological damage of NLRC4^−/−^ mice were significantly impaired. NLRC4^−/−^ macrophages showed a lower release of inflammatory factors, reactive oxygen species (ROS), and lactate dehydrogenase (LDH). Collectively, our results demonstrated that the activation of caspase-1 and downstream cytokines mediated by NLRC4 inflammasome in immune cells during *Cryptococcus* infection can enhance pyroptosis of macrophages, affect the phagocytic ability of macrophages, and inhibit the intracellular parasitism of cryptococcus, eventually reducing the burden of fungi.

## 1. Introduction

Cryptococcus neoformans is an encapsulated yeast that causes disease mainly in immunosuppressed hosts, but the morbidity is also increasing in patients with normal immune function [1, 2]. Cryptococcus infects the body through the inhalation of environmental spores or yeasts that are present in environmental sources, causing cryptococcal meningitis and cryptococcal pneumonia [3]. C. neoformans are responsible for over 180 thousand deaths yearly worldwide [4], which is a serious threat to human health.

RETRACTED

C. neoformans is considered a facultative intracellular pathogen because of its capacity to survive and replicate inside phagocytes, especially macrophages. This ability is heavily dependent on a capsule outside of the cell wall, which is mainly composed of the antiphagocytic glucuronoxylomannan [5]. Cryptococcus can not only resist phagocytosis by macrophages but also survive and even proliferate in cells. Although the virulence of Cryptococcus has nothing to do with its intracellular proliferation rate, the intracellular proliferation rate of Cryptococcus gordonis exceeds that of other pathogenic bacteria.

Cryptococcus neoformans seems to be more likely to establish stable extrapulmonary infections, especially in the central nervous system. Most cases of fulminant meningitis occur in people infected with Cryptococcus neoformans, and only 35% of patients have lung infections, while the same infection is as high as 72% in cases of Cryptococcus gattii. However, the detailed mechanisms for the interaction of C. neoformans with host cells are still poorly studied.

Nucleotide binding and oligomerization domain (NOD)-like receptors (NLR) are cytoplasmic pattern-recognition receptors (PRRs) that play a key role in the innate immune response and can recognize pathogen-associated molecular patterns (PAMP) and damage-related molecular patterns [6]. NLR is subdivided into four subfamilies based on the N-terminal domain, such as the NLR pyridine domain (NLRP), and is related to inflammasome assembly, signal transduction, transcription activation, and autophagy [7, 8]. Recent studies have shown that NLR is related to sensing fungi. After activation, NLR is responsible for apoptosis-related dot-like proteins in macrophages and dendritic cells (DCs) that produce interleukin (IL)-1*β* and IL-18, including caspase recruitment domain (CARD) caspase-1 activation of inflammasomes [9, 10].

The inflammasomes discovered so far include NLRP1, NLRP3, NLRP6, NLRP7, NLRP12, NLRC4, and NLR family member neuronal apoptosis inhibitor protein (NAIP). They are all able to form a classic inflammasome complex containing the adaptor protein apoptosis-associated speck-like protein containing CARD (ASC) and the cysteine protease caspase 1 [11, 12]. In the past 10 years or so, studies have found that the activation of inflammasomes can activate the cysteine aspartate proteolytic enzyme 1 (caspase-1, CASP1) [13], so that the inactive CASP1 precursor (pro-CASP1) is cleaved into active CASP1, thereby promoting the cleavage of inactive IL-1*β* precursors (pro-IL-1*β*) and IL-18 precursors (pro-IL-18) into mature IL-1*β* and IL-18, which are released outside the cell participate in the process of inflammation and injury of the body [13]. Caspase-1 cleaves the precursor cytokines pro-IL-1*β* and pro-IL-18 and the pore-forming protein gasdermin D. The oligomerization of the active fragment of gasdermin D leads to the formation of holes in the cell membrane, triggering pyroptosis [14]. These holes allow the passive release of biologically active IL-1*β* and IL-18 from the cell.

RETRACTED

IL-1*β* and IL-18 have been shown to be essential for optimal activation of the antifungal activity of macrophages [15]. Polymorphisms in the IL-1 gene cluster may be important for susceptibility or resistance to invasive pulmonary aspergillosis in humans. Both IL-1*α* and IL-1*β* have also been shown to play an important role in disseminated candidiasis, and IL-1 signaling has been shown to promote the fight against lung histoplasma and host-resistant coccidioides infection [16, 17].

However, the interaction of cryptococcosis with the host's natural immunity, especially the role of the inflammasome family, has not been fully elucidated. Therefore, it is urgent to explore the role of the inflammasome family in cryptococcal lung infections and the underlying mechanisms. Herein, we explored whether Cryptococcus gattii can activate the inflammasome NLRC4 to release the inflammatory factors interleukin-1*β* and IL-18, and cause pyroptosis, promote the killing of Cryptococcus, and inhibit its intracellular parasitism.

## 2. Materials and Methods

### 2.1. Cryptococcus Culture

The reference strains of *Cryptococcus gattii* R265 (serotype B), GFP-R265, were obtained from F. Robin laboratory. The fungus was kept in a 20% glycerol stock and grown on yeast extract peptone dextrose (YPD) agar plates at 30°C. The liquid culture was grown in YPD medium at 30°C for 20–24 hours in a shaking incubator at 180 rpm. The fungal cells were centrifuged at 2000 g for 2 minutes, washed 3 times, and then resuspended in sterile phosphate buffered saline (PBS). In some experiments, the fungus was heat-inactivated by incubating at 70°C for 1 hour, and after placing it on a YPD agar plate for 2 days, inoculation with inactivated *Cryptococcus gattii* was performed and no growth was observed.

### 2.2. THP-1 Cell Culture

THP-1 cells are stored in RPMI 1640 medium containing 10% FBS, 100 IU/ml penicillin, 1 mg/ml streptomycin, and 50 mM 2-ME at 37°C and 5% CO_2_. To differentiate into macrophages, THP-1 cells were incubated with 100 ng/ml PMA for 3 hours, then washed twice with PBS, and left to stand for 48 hours before use.

RETRACTED

### 2.3. BMDC Preparation

As mentioned above, mouse bone marrow-derived dendritic cells (BMDC) were prepared. In short, bone marrow cells were collected, suspended in PBS by adding RBC lysis buffer to remove red blood cells, and then seeded in 1640 medium at a density of 5 × 10^5^ cells/ml, which contained GM-CSF (20 ng/ml; PeproTech, Rosemont, IL, USA). A humidified incubator containing 5% CO_2_ at 37°C. With the same dose of GM-CSF, change the liquid in half every 3 days. The cells were harvested on the 7th day, and the purity of CD11c + cells tested by flow cytometry was higher than 80%.

### 2.4. WT and NLRC4^−/−^ Mice Preparation

Male specific pathogen-free (SPF) WT and NLRC4−/− mice derived from the C57BL/6N genetic background, 7 to 8 weeks of age, were used in all experiments. The WT mice (60 in total) were purchased from Shanghai SLAC Laboratory Animal Co., Ltd. (Shanghai, China). The NLRC4−/−mice were provided by Dr. Nunez, University of Michigan, and NLRC4−/− mice primer sequence used for identification was as follows: (1) GAAGCCTCAACGGCAACGAGCACTC; (2) GCAGGAATCAATCCAGAGTCTGAG; (3) GCAGCGCATCGCCTTCTATC.

The WT & NLRC4−/− mice care animals were maintained in a SPF facility and monitored daily by veterinary staff. The Ethical Committee of the Department of Laboratory Animal at Shandong University approved all the experiment protocols.

### 2.5. Mouse Serum Collection

To collect mouse serum, WT C57BL/6 mice were anesthetized by injection of 1% sodium pentobarbital, and blood was collected by cardiac puncture. The whole blood was placed in an EDTA anticoagulation tube, and mouse serum was collected by centrifugation at 3000 rpm for 15 minutes at 4°C.

### 2.6. Detection of Total Lung Cytokines and Chemokines

Euthanasia was performed on mice, and the lungs were washed with 10 ml ice-cold PBS. Whole lung protease and phosphatase inhibitor mixture (Fisher Scientific) was homogenized with Halt in 2 ml PBS. Supernatant was collected using sterilized glass tube and rotated at 12,000 rpm for 20 minutes, and store aliquots at −80°C for further analysis. The following cytokines and chemokines in whole lung protein samples were analyzed by ELISA (Thermo Systems, Waltham, MA, USA).

### 2.7. Mouse Model of Fungal Infection

For infection, yeast cells were cultured in YPD medium in a shaking incubator for 24 hours. The culture was then washed in phosphate buffered saline (PBS), counted using a hemocytometer, and resuspended in PBS at a concentration of 2 × 10^6^ yeast cells/ml as previously described. Mice were treated with PBS or infected with Cryptococcus via intranasal vaccination. After anesthesia with isoflurane, each mouse received 50 *μ*l of yeast cell suspension (1.0 × 10^5^ yeast cells/mouse). One day after the infection, the infected mice were euthanized using CO_2_ inhalation. In order to study the kinetics of immune cell infiltration and analyze the expression of chemokines, mice were infected and analyzed on days 1, 7, and 14 after infection. For lung fungal burden analysis, the lungs were homogenized in sterile PBS, diluted, and then inoculated on YPD agar for colony count. After 48 hours of incubation at 30°C, the CFU was calculated. For survival analysis, mice were checked twice a day, and if they looked painful or dying, they were euthanized.

RETRACTED

### 2.8. Tissue Separation and CFU Analysis

After the mice were euthanized with carbon dioxide, their lungs, spleen, and liver were excised and placed in sterile, ice-cold PBS. The tissue is then homogenized using a glass tube, and the pestle is connected to a mechanical tissue homogenizer (Glas-Col) and diluted in SDA. The plate was incubated at 37°C for 72 h.

## 3. Results

### 3.1. Cryptococcal Infection Can Activate the Nod-Like Receptors of Caspase-1 and NLRC4 Inflammasomes in Macrophages and DCs

Since the maturation and secretion of IL-1*β* depend to a large extent on the function of inflammasomes, we set out to investigate whether Cryptococcus can activate inflammasomes in human monocyte-derived macrophages. Compared with other subtypes of Cryptococcus, *cryptococcus gattii* can proliferate in host cells faster than others. We used *cryptococcus gattii R*265 to derive dose-dependent macrophages from THP-1 cells and MHS that induced NLRC4 expression and robust IL-1*β* secretion (Figures 1(a) and 1(b)).

Different types of cells show differences in the activation of inflammasomes. For example, the activation threshold of inflammasomes in mouse macrophages is much higher than in human macrophages. Although we can observe phagocytosis in mouse macrophages, as a facultative intracellular fungal pathogen, Cryptococcus neoformans can replicate in host phagocytes, but the phagocytosis of Cryptococcus induces few cytokines produce. As the most important APC, dendritic cells are much more sensitive than other cells in sensing invading pathogens. This indicates that Cryptococcus neoformans uses specific mechanisms to avoid the activation of inflammasomes in macrophages, which may also be inflammatory in these cells.

As most virulence factors (capsular polysaccharides, lipoproteins) are retained at the temperature used to heat-killing, we used the heat-inactivated *cryptococcus gattii R*265, and checked that the heat-inactivated strains also induced BMDC to secrete IL-1*β* and IL-18 (Figures 1(c) and 1(d)).

RETRACTED

For most inflammasome assemblies, they are able to form a classic inflammasome complex containing the adaptor protein ASC and the cysteine protease caspase 1. NLRC4 can recruit caspase 1 without ASC because of its structure with a CARD domain. We found that the R265 strain of *Cryptococcus gattii* could induce the expression of NLRC4 protein in THP-1 derived macrophages and mouse alveolar macrophages MHS, which is direct evidence for the activation of NLRC4 inflammasomes (Figure 1(e)). In addition, we also found that the *Cryptococcus gattii R*265 strain can activate caspase-1 maturation in macrophages derived from BMDC (Figure 1(f)). At the same time, we used NLRC4 siRNA and control siRNA to knock down the THP-1 cell-derived macrophages, respectively. ELISA detected the downstream IL-1*β* and IL-18 expression changes and found reduction of both IL-1*β* and IL-18 by various degrees (Figure 1(g)). Therefore, the *Cryptococcus gattii R265* strain induces the secretion of IL-1*β* and IL-18 in human and mouse macrophages and activates the inflammasome.

### 3.2. The Survival Rate, Lung Fungal Burden, and Histopathological Damage of NLRC4-/- Mice Were Impaired

We first inoculated yeast cells with GFP-R265 by intrapharyngeal (ip) injection, and then used NLRC4 knockout mice and control mice to construct inhalation models to explore the mechanism of NLRC4 in cryptococcal infection models. We use 10^5 *cryptococcus*, and mice infected with any species begin to die 2 weeks after vaccination. However, NLRC4 KO mice infected with R265 died faster than mice in the control group (Figure 2(d)) (*P*=0.0208). Both groups of mice had a severe lung fungal burden during the infection period, and it can be shown by lung fluorescence values that the fungal burden of NLRC4 KO mice was higher than that of mice in the control group (Figures 2(a) and 2(b)). Next, we used mouse live CT scan and in vitro tissue CT, respectively, and both showed that the lungs of the NLRC4 KO group mice had more cryptococcal nodules and damage than the control group (Figure 2(c)).

One week after inoculation, the lungs of NLRC4 KO mice infected with *R*265 were significantly larger than those of control mice. And its PAS slice also showed that *Cryptococcus* with PAS appeared to be round with a diameter of 5∼15 microns, extracellular, magenta, and yeast-like organisms (Figure 2(e)). PAS staining showed that the average number of PAS positive cells in each lung in the control group was significantly lower than that in the NLRC4 knock out group. In addition, although yeast cells could be recovered from each extrapulmonary organ examined, R265 cells could also be detected in the liver and kidney, but the results for fungal load were similar. These data indicate that R265 can be excreted from the lungs and spread to other organs, but the key to controlling its quantity lies in the lungs.

RETRACTED

### 3.3. NLRC4^−/−^ Macrophages Showed a Lower Release of Inflammatory Factors

When pyroptosis occurs, the cells will release the inflammatory factors interleukin-1*β* and IL-18 when caspase-1 is activated, which will attract more inflammatory cells and aggravate the inflammatory response. At the same time, pores are formed, which allow the release of cytoplasmic contents, such as lactate dehydrogenase (LDH). So, we first verified that the R265 strain can cause caspase-1 activation in macrophages (Figure 3(a)). Then we compared the difference in caspase-1 activation between the control group and the NLRC4 KO group. Caspase-1 is activated in a time-dependent manner, and NLRC4 can significantly affect the expression of caspase-1. Next, we detected the release of reactive oxygen species (ROS) from macrophages by fluorescence microscopy and flow cytometry. The presence of NLRC4 can promote the production of ROS (Figure 3(b)). The LDH presenting in the extracellular media was quantified as a measure of pyroptosis-induced by the inflammasome. Our results show that NLRC4 can affect the release of LDH caused by *Cryptococcus* (Figure 3(c)). We observed that bronchoalveolar lavage fluid (BALF) was collected from cryptococcal-infected mice, and the number of white blood cells in BALF was counted (Figure 3(d)). It was found that there was one white blood cell in the alveolar lavage fluid dominated by alveolar macrophages. We speculate whether NLRC4 caused the pyroptosis of alveolar macrophages, making the number of macrophages decrease. Finally, we verified the effect of NLRC4 on the phagocytosis of macrophages (Figure 3(e)).

## 4. Discussion

*Cryptococcus neoformans* is one of the common conditional pathogenic fungi that exists widely in nature and is divided into *Cryptococcus neoformans var. neoformans* and *Cryptococcus neoformans var. gattii* [18]. Both Cryptococcus neoformans and Cryptococcus gattii can cause cryptococcal pneumonia and cryptococcal meningitis, but Cryptococcus gattii tends to cause cryptococcal pneumonia rather than meningitis. It has also been reported that, compared with Cryptococcus neoformans variants, Cryptococcus gattii can induce higher concentrations of proinflammatory related factors, such as IL-1*β*, IL6, and Th17/22 related cytokines. In addition, the clinically isolated Cryptococcus gattii can also induce higher cytokines [19].

Inflammasomes are high-molecular weight complexes formed in the cytosol of a cell that serve as a platform for inflammatory caspase activation. In addition to activating the release of cytokines, inflammasomes can sense microbial infection or host cell damage and trigger the production of cytokines and a form of proinflammatory cell death called pyroptosis [14]. In the process of cell pyroptosis, under the stimulation of external conditions, the precursor of caspase-1 can form a polymer complex with the pattern-recognition receptors NLRP1, NLRP3, NLRC4 [20], etc. through the adaptor protein ASC, the inflammasome, also known as the dependent caspase-1 inflammasome. When caspase-1 is activated, cells will release the inflammatory factors interleukin-1*β* (IL-1*β*) and IL-18, which will attract more inflammatory cells and aggravate the inflammatory response. Pores are formed when pyroptosis occurs, which allows the release of cytoplasmic contents such as LDH and inflammatory cytokines [21].

RETRACTED

In this study, we found that *Cryptococcus gattii* can better activate the NLRC4 inflammasome and significantly affect the activation of downstream caspase-1 and the expression of related cytokines, which indicates that *Cryptococcus* gattii was directly or indirectly recognized by the host through NLRC4 (Figure 4). Previously, it was reported that the capsular mutant *Cryptococcus cap*59Δ can activate the ability of the NLRP3 inflammasome [22, 23]. This indicates that *Cryptococcus* capsules directly or indirectly prevent the passage of NLRP3 that would otherwise recognize fungi. *Cryptococcus* mainly infects population with suppressed immunity and mainly causes lung infection. There are significant differences between *Cryptococcus neoformans* and *Cryptococcus gattii* in terms of prevalence, pathogenicity, symptoms, diagnosis, and treatment. These differences in NLRC4 are of great significance for the prevention and treatment of *cryptococcus* and the prognosis of infection.

Our in vivo data show that during lung infection with *Cryptococcus gattii R*265, the infiltration of leukocytes into the lungs and the clearance of fungi depend on the NLRC4 inflammasome. And since *Cryptococcus* is a facultative intracellular pathogen, the intracellular recognition of this pathogen is very important for elimination. Proper pyroptosis can inhibit the intracellular parasitic process of Cryptococcus. Our data indicate that NLRC4 affects the release of caspase-1, LDH, and ROS and the process of macrophage phagocytosis, which indicates that the inflammasome NLRC4 may be involved in the cell death process of cryptococcal infection when pyroptosis is mediated. This will be an interesting and important topic for future research.

RETRACTED

So far, the control of *Cryptococcus* is still challenging, especially in patients with weakened immune functions. Although some animal studies have found that the Th1 and Th17-cell responses are protected, while the Th2 response is harmful, the activation of inflammasomes can affect different balanced T helper cell responses [24]. On one hand, these immune responses are important for clearing cryptococcal infections. On the other hand, overwhelming inflammation can also cause harmful effects. Our current research shows that the host's NLRC4 inflammasome recognizes *Cryptococcus* gattii, thus indicating the importance of NLRC4 in identifying and controlling cryptococcal infections. Although inflammasome activation may also lead to harmful results, such as tissue damage, it is appropriate to conclude that activating the function of the NLRC4 inflammasome may be a new method to control cryptococcosis.

The inflammasome has become an important platform, responsible for the proteolytic processing of the inflammatory cytokines IL-1*β* and IL-18 and pyrolysis. Although many pathogens have been found to activate inflammasomes, fungal pathogens that activate inflammasomes have not been extensively studied. C. gattii is an important fungal pathogen, and the interaction between host cells and C. gattii is unclear. Importantly, and in addition to the reported NLRP3, we found that C. gattii can also activate the caspase-1 inflammasome NLRC4 and play a certain role in the process of antifungal host immunity, especially in macrophages and DC cells, which represented the innate immunity stage.

Nonetheless, there may be some possible limitations in this study that could be addressed in future research, such as the mechanism of NLRC4 regulating the activation of casepase-1 has not been studied deeply enough, and the specific signaling pathway and binding site have not been confirmed. Does the activation of the NLRC4 inflammasome affect the efficacy of antifungal drugs against pulmonary Cryptococcus infection? This needs further experimental verification.

## 5. Conclusions

Our results suggest that NLRC4 can affect the release of key cytokines by DCs and macrophages. IL-1*β* and IL-18 are key cytokines that activate and control inflammatory bodies and play an important role in host resistance to cryptococcal infection. In addition, NLRC4 affects the pyroptosis of macrophages. Proper pyroptosis can inhibit the intracellular parasitic process of Cryptococcus and help the body eliminate Cryptococcus. The activation of the NLRC4 inflammasome is of great significance for the prevention and treatment of Cryptococcus and the prognosis after infection.

RETRACTED

## Figures and Tables

**Figure 1:** Internalized *Cryptococcus* activates the NLRC4 inflammasome, thereby activating caspase-1-related IL-1*β* and IL-18 secretion. (a) NLRC4 mRNA expression in THP-1 cell-derived macrophages were infected with the yeast form of *cryptococcus* at the indicated MOI for the indicated time. (b) IL1-*β* mRNA expression in THP-1 cell-derived macrophages were infected with the yeast form of *cryptococcus* at the indicated MOI for the indicated time. (c) Different ratios of *Cryptococcus* were used to stimulate BMDC cells, and IL-1*β* and IL-18 in the supernatant were determined by ELISA. (d) The THP-1 cell-derived macrophages and MHS cells were stimulated with *Cryptococcus* for 2 hours, and the expression levels of IL-1*β* mRNA and IL-18 were measured by real-time PCR. (e) WB was used to detect the activation of NLRC4 protein by *Cryptococcus* in THP-1 and BMDC cells, respectively. (f) Detection of caspase-1 activation by *Cryptococcus* in BMDC. (g) Use NLRC4 siRNA and Control siRNA to knock down BMDC, respectively, and detect the expression changes of downstream IL-1*β* and IL-18 by ELISA.

**Figure 2:** NLRC4 affects the fungal burden and survival rate of mice. NLRC4 is required for survival and control of fungal burden after infection with Cryptococcus gattii GFP-R265. Wild-type (WT) and NLRC4-deficient (NLRC4^−/−^) mice were infected intratracheally with 10^5^ CFU of Cryptococcus gattii R265. (a, b) The chest cavity of mice was exposed to the fluorescence camera, and the lung fluorescence imaging was performed. The fluorescence intensity represented the amount of fungal load. (b) As the average fluorescence intensity. (c) Lung scan imaging of WT and NLRC4^−/−^ mice using Micro CT, representative image. (d) Mice were observed for up to 30 days for survival analysis (*n* = 10 mice/strain, using a log-rank test). (e) Significant reduction of inflammation in NLRC4−/−compared to WT mice; Mucicarmine staining shows numerous heavily encapsulated extracellular Cryptococcus gattii in the airspaces of NLRC4−/− mice compared to WT mice. Representative images of lungs stained with PAS. (f) Fungal burden in the lung, liver, and spleen at serial time intervals was determined by plating tissue homogenates on Sabouraud dextrose agar. CFU data are shown as mean ± SEM and representative of two independent experiments (*n* = 4 mice/strain/time point). ^*∗*^*P* ≤ 0.05, ^*∗∗*^*P* ≤ 0.01, and ^*∗∗∗*^*P* ≤ 0.01. (g) Detection of cytokines in mouse lung tissue grinding fluid by ELISA.

**Figure 3:** NLRC4 is required for Cryptococcus-mediated casepase-1 activation and pyroptosis. Peritoneal macrophages were plated at 5 × 10^5 cells/well and treated withR265, LPS. Cells were washed, lysed, (a) and 100 *μ*g of lysates were assayed using Caspase-1 assay kit (ab39412).PBS was used as a control. (b) ROS was measured by staining the Peritoneal macrophages with DCFDA cellular ROS detection assay kit according to the manufacturer's instructions. ROS generation was observed under a fluorescence microscope at 200*x* magnification (left). ROS generation was analyzed by flow cytometry (right). (c) Pyroptosis was assessed by measuring LDH release in the supernatant. (d) Mouse BALF cell number of WT & NLRC4-/-. (e) Peritoneal macrophages from WT and NLRC4-/- mice were incubated with GFP-R265 for 6 hours, and phagocytosis was detected by flow cytometry. ^*∗*^*P* ≤ 0.05 5, ^*∗∗*^*P* ≤ 0.01, and ^*∗∗∗*^*P* ≤ 0.01.

RETRACTED

**Figure 4:** NLRC4 resists cryptococcal infection in the lungs of mice by activating caspase-1 mediated release of IL-*β* and IL-18 and appropriate pyroptosis.

## Data Availability

The datasets used and analyzed during the current study are available from the corresponding author on reasonable request.

## References

[1] Barreto-Bergter E., Figueiredo R. T. (2014). Fungal glycans and the innate immune recognition. *Frontiers in Cellular and Infection Microbiology*.

[2] Ydens E., Amann L., Asselbergh B. (2020). Profiling peripheral nerve macrophages reveals two macrophage subsets with distinct localization, transcriptome and response to injury. *Nature Neuroscience*.

[3] Giladi A., Wagner L. K., Li H. (2020). Author Correction: cxcl10+ monocytes define a pathogenic subset in the central nervous system during autoimmune neuroinflammation. *Nature Immunology*.

[4] Rajasingham R., Smith R. M., Park B. J. (2017). Global burden of disease of HIV-associated cryptococcal meningitis: an updated analysis. *The Lancet Infectious Diseases*.

[5] Crawford C. J., Wear M. P., Smith D. F. Q. (2021). A glycan FRET assay for detection and characterization of catalytic antibodies to the Cryptococcus neoformans capsule. *Proceedings of the National Academy of Sciences*.

[6] Heung L. J., Hohl T. M. (2019). Inflammatory monocytes are detrimental to the host immune response during acute infection with Cryptococcus neoformans. *PLoS Pathogens*.

[7] Pandey A., Ding S. L., Qin Q.-M. (2017). Global reprogramming of host kinase signaling in response to fungal infection. *Cell Host & Microbe*.

[8] Su S.-H., Wu Y.-F., Lin Q., Wang D.-P., Hai J. (2019). URB597 protects against NLRP3 inflammasome activation by inhibiting autophagy dysfunction in a rat model of chronic cerebral hypoperfusion. *Journal of Neuroinflammation*.

[9] Wong S. S. W., Aimanianda V. (2017). Host soluble mediators: defying the immunological inertness of Aspergillus fumigatus conidia. *Journal of Fungi*.

RETRACTED

[10] Portnoy J. M., Williams P. B., Barnes C. S. (2016). Innate immune responses to fungal allergens. *Current Allergy and Asthma Reports*.

[11] Kay C., Wang R., Kirkby M., Man S. M. (2020). Molecular mechanisms activating the NAIP‐NLRC4 inflammasome: implications in infectious disease, autoinflammation, and cancer. *Immunological Reviews*.

[12] Howrylak J. A., Nakahira K. (2017). Inflammasomes: key mediators of lung immunity. *Annual Review of Physiology*.

[13] Pinkerton J. W., Kim R. Y., Robertson A. A. B. (2017). Inflammasomes in the lung. *Molecular Immunology*.

[14] Jang Y., Lee A. Y., Jeong S.-H. (2015). Chlorpyrifos induces NLRP3 inflammasome and pyroptosis/apoptosis via mitochondrial oxidative stress in human keratinocyte HaCaT cells. *Toxicology*.

[15] Yashiro T., Yamamoto M., Araumi S. (2021). PU.1 and IRF8 modulate activation of NLRP3 inflammasome via regulating its expression in human macrophages. *Frontiers in Immunology*.

[16] Swaminathan N., Vinicius J. M., Serrins J. (2020). Hemophagocytic Lymphohistiocytosis (HLH) in a patient with disseminated histoplasmosis. *Case reports in hematology*.

[17] Viriyakosol S., Walls L., Okamoto S., Raz E., Williams D. L., Fierer J. (2018). Myeloid differentiation factor 88 and interleukin-1R1 signaling contribute to resistance to coccidioides immitis. *Infection and Immunity*.

[18] Mukaremera L., McDonald T. R., Nielsen J. N. (2019). The mouse inhalation model of cryptococcus neoformans infection recapitulates strain virulence in humans and shows that closely related strains can possess differential virulence. *Infection and Immunity*.

[19] Hansakon A., Ngamskulrungroj P., Angkasekwinai P. (2020). Contribution of laccase expression to immune response against cryptococcus gattii infection. *Infection and Immunity*.

[20] Wang S., Qing D. (2020). Progress in inflammasome activation and pyrolysis in alcoholic liver disease. *Zhong nan da xue bao. Yi xue ban = Journal of Central South University. Medical sciences*.

[21] Burgel P., Marina C., Saavedra P. (2020). Cryptococcus neoformans secretes small molecules that inhibit IL-1beta inflammasome-dependent secretion. *Mediators of Inflammation*.

[22] Duncan J. A., Canna S. W. (2018). The NLRC4 inflammasome. *Immunological Reviews*.

[23] Guo C., Chen M., Fa Z. (2014). Acapsular Cryptococcus neoformans activates the NLRP3 inflammasome. *Microbes and Infection*.

[24] May R. C., Stone N. R. H., Wiesner D. L., Bicanic T., Nielsen K. (2016). Cryptococcus: from environmental saprophyte to global pathogen. *Nature Reviews Microbiology*.

